# Moisture Impact on Static and Dynamic Modulus of Elasticity in Structural Normal-Weight Concretes

**DOI:** 10.3390/ma17153722

**Published:** 2024-07-27

**Authors:** Lucyna Domagała, Maria Margańska, Marek Miazgowicz

**Affiliations:** Faculty of Civil Engineering, Cracow University of Technology, 31-155 Kraków, Poland; maria.marganska@doktorant.pk.edu.pl (M.M.); marek.miazgowicz@doktorant.pk.edu.pl (M.M.)

**Keywords:** structural concrete, normal-weight aggregate, moisture content, density, ultrasonic pulse velocity, compressive strength, modulus of elasticity

## Abstract

In the case of concrete built into a structure, the static secant modulus of elasticity (*E_c,s_*) is often estimated based on its dynamic value (*E_d_*) measured by the ultrasonic pulse velocity method instead of direct tests carried out on drilled cores. Meanwhile, the prevailing equations applied to estimate *E_c,s_* often overlook the impact of concrete moisture. This study aimed to elucidate the moisture impact across two normal-weight structural concretes differing in compressive strength (51.6 and 71.4 MPa). The impact of moisture content was notably more evident only for the weaker concrete, according to dynamic modulus measurements. In other cases, contrary to the literature reports and expectations, this effect turned out to be insignificant. These observations may be explained by two factors: the relatively dense and homogeneous structure of tested concretes and reduced sensitivity of *E_c,s_* measurements to concrete moisture condition compared to *E_d_* measurements obtained using the ultrasonic method. Additionally, established formulas to estimate *E_c,s_* were verified. The obtained modulus results tested under different moisture conditions of normal-weight concretes were also compared with those of lightweight aggregate concretes of identical volume compositions previously obtained in a separate study.

## 1. Introduction

To design concrete members and structures, it is necessary to know the value of the concrete modulus of elasticity, which is its critical mechanical property. The value of this characteristic is essential for calculating stress–strain relationships, deflection of structural members, crack width, prestress force losses, and stresses resulting from environmental strains. Nevertheless, the values provided in the European Standard EN-1992-1-1 [1] for designing concrete structures should be considered only as general guidelines. Despite the fact that modulus value is influenced by various parameters, including the type and proportion of concrete constituents, the condition of the concrete, and the testing methodology used, the standard EN-1992-1-1 [1] considers only the influence of concrete compressive strength and, to some extent, the type of aggregate within certain limits. Many types of aggregates commonly used in structural concretes (e.g., granite) have not been accounted for in this approach. Moreover, many publications (e.g., [2,3,4,5,6]) have shown that due to the diverse properties of a given type of aggregate depending on its source, considering the aggregate effect on the modulus value solely based on its type is inappropriate.

Therefore, it is recommended to specifically test the modulus if a structural element is susceptible to variations from these standard values. It should also be noted that the existing European Standard dedicated to determining the concrete modulus of elasticity, EN 12390-13 [7], does not specify the influence of various technical parameters, including the specimen type, its dimensions and shape, as well as the method applied (Method A or Method B). However, the research results reported in [8,9] indicate that these factors can, in some cases, affect the modulus value to a greater extent than material factors. Another issue is the effect of moisture content on the determined value of the concrete modulus. While the standard EN 12390-13 [7] requires saturation of concrete specimens in water before modulus testing, in practice, cores taken from structures often do not meet this requirement, and they are tested in their natural state, as received after drilling. The same problem applies to testing concrete built into structures using non-destructive methods, such as the popular ultrasonic pulse-velocity method.

Meanwhile, based on the few studies conducted on this subject, it emerges that the moisture content of concrete is a parameter that may considerably influence the modulus, yet it is often overlooked. Unlike the extensive studies on how moisture affects concrete’s compressive strength (e.g., [2,3,4]), research on its impact on the modulus of elasticity is rather scarce. Contrary to compressive strength, where increased moisture content typically reduces strength, the modulus of elasticity can increase if the concrete moisture content surpasses a given value relative to concrete water absorption [4,10,11]. The static modulus of elasticity (*E_c,s_*) specified on specimens fully saturated with water has been 3% to 55% higher compared to the modulus determined on specimens in dry conditions [10,11,12,13,14]. The above increase seems to be dependent on concrete porosity and composition. As demonstrated in references [11,12,13], for normal-weight concretes the characteristic range of increase in *E_c,s_* when specified on wet specimens was 12% to 32% compared to dry specimens. This increase is attributed to the reduced material deformability when the water fills its pores.

However, research [15] has shown that concrete drying may cause a reduction in the modulus of elasticity, owing to cracks forming from different shrinkages of cement matrix and aggregate. That is why, in the case of composites with bigger and stiffer aggregates, a more pronounced modulus reduction has been observed. Some studies (e.g., [11,16]) also suggest an inverse relationship between concrete strength and modulus of elasticity with moisture content, although these studies often involve testing at higher temperatures and non-standard methods.

The influence of concrete moisture content also proved to be significant in dynamic modulus testing (*E_d_*). This issue is particularly significant given that in many technical studies, the static modulus of elasticity is not directly measured but estimated on the basis of the *E_d_* value. According to reference [17], pulse velocity is considerably affected by both the mean moisture content and its deployment. The extent of pore filling with liquid and crack length also play important roles.

While it is generally assumed that the relationships between static modulus of elasticity and dynamic modulus of elasticity are unaffected by the curing method, air entrainment, cement type, or test conditions [4,18], the findings presented in [19] suggest that the relationships between *E_d_* and *E_c,s_* may vary depending on the moisture condition of concrete. However, this hypothesis requires validation through further research, as the concrete described in [19], despite having the same composition, exhibited notably different mechanical properties and microstructure caused by distinct curing. Certain support for the above hypothesis is provided in the results of tests conducted on lightweight concretes, reported in [14]. In the case of these concretes, regardless of their strength level, the impact of the moisture content on *E_d_* was much more pronounced than its influence on *E_c,s_*. Nevertheless, it should be noted that due to the specific nature of lightweight concretes and their significantly higher porosity, moisture content’s impact on measurements of the modulus of normal-weight concretes may differ.

The basic objective of this study was to investigate how the moisture content of structural normal-weight concrete affects the values of modulus of elasticity, determined dynamically using the non-destructive ultrasonic pulse velocity method, and statically under cyclic loading at compression. A further goal was to examine the relationship between these two types of moduli. It was also important to compare the obtained results for normal-weight concretes with the results reported in [14] reached by lightweight concretes made from the same ingredients, except for the coarse aggregate, which was cured and tested in the same way.

## 2. Materials and Methods

Two series of normal-weight structural concretes were prepared for the tests. Exactly as in the case of the lightweight concrete series described in [14], both normal-weight concrete series maintained comparable volumes of coarse aggregate (ca 45%) and mortar–cement matrix (ca 55%). Since two different water–cement ratios (w/c), 0.37 and 0.55, were used, these two composites reached various levels of mechanical properties. Additionally, to provide a constant consistency for both concrete mixtures, a superplasticizing admixture was dosed to the fresh concrete with the lower water–cement ratio. The following constituent materials were used for both concrete series: tap water, cement CEM I 42.5 R, 0/2 mm natural sand, and 4/16 mm natural gravel. The coarse aggregate consisted of a blend of single-crushed rounded aggregates with predominantly sandstone grains (Figure 1).

The key properties of the coarse aggregate fraction were as follows: the particle density was 2650 kg/m^3^ (acc. to EN 1097-6 [20]); the bulk density was 1730 kg/m^3^ (acc. to EN 1097-3 [21]); the 24 h water absorption was 1.5% (acc.to EN 1097-6 [20]).

Table 1 presents the contents of constituent materials used to make both normal-weight concretes.

Twenty-one standard cylindrical specimens (with a diameter of 150 mm and a length of 300 mm) were cast for each concrete series. After 24 h, all specimens (42) were demolded and stored for 28 days in water at 20 °C in accordance with EN 12390-2 [22]. Then, the specimens were removed from water and some of them were tested for the standard age of 28 days. The rest of the specimens were kept in air at 20 °C and relative humidity of 50% for the next three years. The curing conditions for both test ages are presented in Figure 2.

To classify the concretes, their density and strength were specified at the standard age of 28 days. Additionally, the tests of static secant modulus of elasticity were carried out at this time. Nevertheless, the main modulus tests were to be conducted after 3 years. Such a long time of curing before testing aimed to eliminate the impact of time on the determined values of both moduli: *E_d_* and *E_c,s_*. Table 2 contains the details of the research program, including the test type, the standard procedure, as well as the age and number of standard cylinders prepared for each concrete series.

For 28 days, mechanical properties were tested on specimens saturated with water as was recommended in EN 12390-13 [7] and EN 12390-3 [24]. However, the 28-day density was determined sequentially in two moisture states: initially in a water-saturated condition, followed by a dry condition. Both density results were used to estimate the water absorption of the concretes.

At the age of 3 years, both physical and mechanical properties were tested initially in air-dry/as-received conditions. After tests in air-dry conditions, the concrete cylinders were placed into water for the next two months. When the specimens reached a constant mass, they were tested again under saturated conditions. Additionally, to check the water absorption after 3 years, 3 specimens, remaining after tests of water-saturated density, were dried out to determine their oven-dried density as well.

The range of stress for *E_c,s_* determination was established on the basis of mean compressive strength (*f_cm, cyl_*). According to Method B included in EN 12390-13 [7], the lower stress *σ_b_* was set to a value 0.13 *f_cm, cyl_* from the standard range (0.10–0.20) *f_cm, cyl_*, while the upper-stress *σ_a_* was set to 1/3 *f_cm, cyl_*. The stress ranges in which both series of concretes were tested, determined on the basis of compressive strength tests, were given in Section 3.2.1. Figure 3 shows loading cycles according to the standard and exemplary cycles recorded during a test of a certain specimen.

To calculate the static stabilized modulus of elasticity, Equation (1) from EN 12390-13 [7] was implemented.

(1) $$E_{c,s\;}=\frac{\sigma_{a}^{m}-\sigma_{b}^{m}}{\varepsilon_{a,3}-\varepsilon_{b,2}}$$

where

- $\sigma_{a}^{m}$—the upper stress measured during the third cycle;
- $\sigma_{b}^{m}$—the lower stress measured during the third cycle;
- *ε_a_*_,3_—the strain corresponding to the upper stress at the third cycle;
- *ε_b_*_,2_—the strain corresponding to the lower stress at the third cycle.

The ultrasonic pulse velocity measurements were carried out directly after static modulus tests according to the method outlined in EN 12504-4 [25]. To calculate the dynamic modulus of elasticity, Equation (2) from ASTM C 215 [26] was followed.

(2) $$E_{d}=\frac{V^{2}D(1+\nu )(1-2\nu )}{\left(1-\nu \right)}.$$

where

- *V*—the ultrasonic pulse velocity measured during the test;
- *D*—concrete density;
- *ν*—concrete Poisson’s ratio of the concrete, taken as 0.2.

EN 12504-4 [24] indicates that ultrasonic velocity may decrease with longer path lengths due to concrete heterogeneity. Therefore, the probes were positioned on both bases of concrete cylinders along their length, which was the least favorable position with the path length of ca 300 mm. Approximately 30 pulse velocity measurements were taken at each probe position to calculate the average value.

Figure 4 illustrates the testing apparatus used for static secant modulus determination, while Figure 5 shows the testing apparatus used for ultrasonic pulse velocity measurements.

To reduce the impact of the structural diversity of concrete on the measurements of dynamic and static moduli, the tests were conducted consecutively on the same set of specimens under varying moisture conditions. This procedure might be accepted as the maximum load used during the mechanical tests was remarkably smaller than the limit of concrete fatigue strength. The results reported in [2,3,4] indicated that the test results are not influenced by subjecting concrete to repeated loads below this limit. However, before conducting the actual tests, it was verified on selected specimens whether the considered normal-weight concretes also did not show the effects of repeated loading. In the case of these concrete specimens, the static modulus of elasticity was tested twice at different locations of sensors on a cylinder side. The results of repeated modulus tests are presented and discussed in Section 3.2.1.

## 3. Results

### 3.1. Initial Tests

The mean values of basic properties of both concrete series, determined at 28 days: compressive strength (***f_cm_***), static secant modulus of elasticity (***E_c,s_***), density in wet condition (*D_w_*), and density in oven-dry conditions (*D_d_*), are presented in Table 3.

The standard deviations for compressive strength were 1.5 MPa for NC1 and 1.0 MPa for NC2, while the standard deviations for modulus of elasticity were 0.3 GPa for NC1 and 0.7 GPa for NC2. In the case of density measurements, none of the individual results deviated from the average value by more than 20 kg/m^3^.

### 3.2. Actual Tests

The mean values of basic properties of both concrete series, determined at the age of 3 years: compressive strength (***f_cm_***), density in air-dry conditions (*D_ad_*), density in wet conditions (*D_w_*), and density in oven-dry conditions (*D_d_*), are presented in Table 4.

The standard deviations for compressive strength tested in standard wet conditions were 1.3 MPa for NC1 and 1.6 MPa for NC2. In the case of density measurements, none of the individual results deviated from the average value by more than 10 kg/m^3^.

The above density test results were used to determine the moisture content and water absorption of the tested concretes. The air-dry series NC1 and NC2 were characterized by moisture content of 1.4% and 0.4%, respectively. Meanwhile, their corresponding water absorption was 5.4 and 2.2%.

Figure 6 demonstrates fracture patterns which were observed after the tests of cylinders of both concrete series after their compression failure. The failure form of cylindrical specimens, visible in Figure 6a, corresponds to the correct forms in accordance with EN 206. Both concretes revealed homogenous structures and a lack of segregation. Furthermore, in spite of coarse aggregate primarily consisting of rounded grains, the tested concretes exhibited relatively good bonds between aggregate and mortar (see Figure 6b). For this reason, cracks propagated both through the bond, as well as through the aggregate grains themselves.

#### 3.2.1. Tests of *E_c,s_*

The stress range *σ_b_*–*σ_a_* in which the concrete cylinders were cyclically loaded to specify static secant stabilized modulus, calculated as described in Section 2, was as follows: 6.5–17.2 MPa for series NC1 and 9.3–23.8 MPa for series NC2.

Table 5 contains the results of *E_c,s_* specified for both dried and wet specimens. The corresponding results of compressive strength measured on wet cylinders used previously for moduli tests were also given in this table. The average *E_c,s_* measured for dried specimens was 30.3 GPa for NC1 and 34.6 GPa for NC2. Meanwhile, the tests carried out on wet cylinders indicated the following results: 29.9 GPa for NC1 and 33.4 GPa for NC2. The moduli standard deviations were in the range of 0.3–0.6 GPa.

Repeated tests of the modulus on saturated cylinders designated as NO. 3 of each concrete series clearly proved the excellent repeatability of the results and lack of impact of subsequent loading cycles on the *E_c,s_* value.

#### 3.2.2. Tests of *E_d_*

Table 6 contains the results of ultrasonic pulse velocity (*V*) measurements specified on both dried and wet specimens. The average velocity measured on dried specimens was 4005 m/s for NC1 and 4181 m/s for NC2. Meanwhile, the tests carried out on wet cylinders indicated the following results: 4311 m/s for NC1 and 4203 m/s for NC2. The velocity standard deviations were in the range of 33–44 m/s.

Table 7 presents the results of dynamic moduli estimations calculated on the basis of Equation (2). The calculations used the oven-dry density as a parameter characterizing the structure of the material. For dried cylinders, the average dynamic moduli were 32.1 GPa for NC1 and 36.0 GPa for NC2. Meanwhile, the tests carried out on wet cylinders indicated the following results: 37.1 GPa for NC1 and 36.4 GPa for NC2. The moduli standard deviations were in the range of 0.4–1.2 GPa.

Figure 7 illustrates some relationships for the measured ultrasonic pulse velocities and estimated dynamic moduli. In the figure, besides the estimations of the dynamic modulus considering the concrete density under the dry condition (marked with a solid line), additional dependencies are presented, taking into account the current concrete density in the state in which it was tested (dashed line). As can be seen from the comparison, consideration of the moisture content of composites in different conditions significantly affects the estimated *E_d_* value. In particular, differences are noticeable when testing specimens saturated in water. However, regardless of the type of density considered in the calculations (oven-dry or current), similarly to the relationships observed for sibling lightweight concretes discussed in [14], it is evident that these relationships are influenced by both the type of concrete and the moisture condition. The impact of the moisture condition appears to be more pronounced. However, this factor is not explicitly included in Equation (3).

For further comparative analysis, the dynamic modulus of elasticity based on Equation (2), considering the density in the oven-dry condition as a relevant indicator of material structure, was taken into account. Incorporating the estimates of *E_d_* based on current density, which is often used in practice, leads to an overestimation of the modulus value due to the double consideration of moisture’s influence (through ultrasonic pulse velocity and density).

## 4. Discussion

As anticipated, different water–cement ratios for both concretes led to notable variations in all physical and mechanical properties. Consequently, based on standard EN-206 [27], concrete NC1 falls within the strength class C 35/45, whereas NC2 qualifies as C55/67.

Both concretes exhibited significant development of mechanical properties for the entire duration of the study. The average 3-year compressive strength of both tested composites was 20% higher compared to the strength measured after 28 days. This strength increase is considered typical for structural normal-weight concretes [2,3,4]. During this time, the static modulus also developed its value noticeably. *E_c,s_* tested on wet specimens increased by 20% for NC1 and 11% for NC2. Comparison of the static modulus values specified in tests with their estimations according to EN 1992 [1], considering the type of coarse aggregate, shows satisfactory convergence.

Figure 8 and Figure 9 present the compilation of all moduli measurement values (*E_c,s_* and *E_d_*) carried out at the age of 3 years on dried and wet specimens for NC1 and NC2, respectively.

### 4.1. Correlation for E_c,s_ and E_d_

Contrary to expectations, the dynamic modulus of elasticity was found to be significantly higher than the static modulus only in the case of NC1 concrete. This trend is particularly noticeable for water-saturated specimens, where the ratio *E_c,s_/E_d_* was 0.81, while for specimens in the air-dry conditions, the corresponding ratio was visibly higher at 0.95. In the case of stronger concrete NC2, *E_c,s_/E_d_* was 0.92 and 0.96 for water-saturated and air-dry conditions, respectively. It is worth noting that the ratio calculated for individual dried specimens was in the range 0.91–0.99, while for wet specimens, it changed from 0.79 to 0.95. These ranges are too broad, and the mean ratios are too high to consider Equation (3) as universal and reliable.

(3) $$E_{c,s\;}=0.83\;E_{d}$$

Equation (3), proposed by Lydon and Balendran [4], is deemed as the most popular and the simplest formula used to assess concrete secant static modulus following its dynamic value. For the tested concretes, except for NC1 in the water-saturated state, its application would lead to a significant underestimation of *E_c,s_* up to 5 GPa. However, in the case of this research, another popular Equation (4) proposed by Swamy and Popovics [4] offers significantly better accuracy (underestimation up to 1 GPa), except for concrete NC1 tested in the water-saturated condition (overestimation up to 5 GPa).

(4) $$E_{c,s\;}=1.04\;E_{d}-4.1$$

A few publications [28,29,30,31,32,33,34] that provide test results of both *E_c,s_* and *E_d_* (measured by the ultrasonic method), indicate that relationships (3) and (4) can lead to even larger differences in estimating *E_c,s_* (up to 17 GPa). The analysis of differences between obtained and estimated static moduli from these tests and the literature data reveals that the correlation between *E_d_* and *E_c,s_* depends on the concrete’s moisture content, as well as the concrete’s structural uniformity. At the given moisture content, a less uniform composite structure (caused by poor adhesion of cement paste to aggregate, or their considerably different stiffness) results in a lower *E_c,s_*/*E_d_*. The tested normal-weight concretes, particularly the stronger concrete NC2, revealed ratios significantly higher than those resulting from data reported in [28,29,30,31,32,33,34] due to their better structural homogeneity, confirmed by high strength and the manner of failure.

### 4.2. The Impact of Water Content in Tested Concretes on Their Moduli Values

Contrary to expectations, the impact of water contained in concrete was found to be significant only in the case of the dynamic modulus and only for the weaker composite NC1. For this concrete, the dynamic modulus based on ultrasonic pulse velocity measured on wet specimens was on average 16% higher than the modulus determined on dried cylinders. However, in the case of the static modulus of elasticity, this effect should be considered negligible. On average, the modulus measured in the saturated state was up to 1% lower than in the dry state. In this case, for individual specimens, the differences in the values of the modulus determined in various moisture conditions reached a maximum of 0.9 GPa, which is less than the scatter observed in the test results. For stronger, less porous concrete, the impact of specimen moisture content proved to be statistically insignificant both in terms of dynamic and static moduli. The fact that NC2 did not show any increase in *E_d_*, even when saturated, may be explained by the more than twofold lower water content in the structure of this concrete (approximately 50 kg/m^3^) compared to more porous concrete NC1 (approximately 120 kg/m^3^).

The results obtained, in relation to those reported in [10,11,12,13,14] regarding the impact of water contained in composites on their modulus of elasticity, broaden the scope of this influence to include cases where such an effect is not observed. In this study, it was confirmed that the occurrence of the moisture content’s impact on concrete modulus, as well as the magnitude of this effect, depend on the type of cement composite, particularly its structural homogeneity and pore structure, as well as the type of test. This research and analysis of literature data unequivocally indicate that the ultrasonic method used for *E_d_* determination seems to be markedly more sensitive to the moisture influence compared to the cyclic loading method used for *E_c,s_* determination. As a result, estimating the standard static secant modulus value (which is intended to be determined in the saturated condition), based on ultrasonic pulse velocity measurements in a composite that is not saturated, can lead to a significant underestimation of the results.

In Figure 10, average moduli test results obtained for structural normal-weight concretes are presented alongside results reported in [14] for structural lightweight concretes with the same volume composition and differing only in the type of coarse aggregate used. From the comparative analysis of modulus values obtained for both types of concretes, it is evident that while the coarse aggregate type has a crucial impact on the static secant modulus, its effect on the dependence of modulus values on concrete moisture is marginal. Owing to the high water absorption of lightweight aggregate used in [14], the water absorption of concretes made with this aggregate was considerably higher (10.1% and 7.9%) than that of corresponding normal-weight concretes (5.4% and 2.2%). Despite the different moisture content of saturated concretes of both types, no significant influence of moisture on *E_c,s_* values was observed in any lightweight or normal-weight concrete. However, during dynamic modulus testing, water contained in both cement paste and aggregate pores contributes to the increase in ultrasonic pulse velocity. As a result, the lightweight concretes discussed in [14] showed an even greater influence of water saturation on the increase in dynamic modulus values compared to the tested normal-weight concretes.

## 5. Conclusions

The carried-out test program did not demonstrate, as was expected, substantially greater dynamic modulus results in comparison to the static one. The only exception was concrete NC1 tested in the water-saturated condition, where the ratio of *E_c,s_/E_d_* was 0.81. For the remaining cases, this ratio ranged from 0.92 to 0.96, which is much higher than 0.83 assumed in the equation proposed by Lydon and Balendran [4].

The research proved the impact of water content only during dynamic modulus testing and only for the weaker, more porous concrete NC1. In this case, *E_d_* under the water-saturation condition was, on average, 16% higher than the value determined on air-dried specimens. In the case of concrete NC2, which has a denser structure and was unable to accumulate the same amount of water as NC1, no impact of specimen moisture on *E_d_* was observed. However, during static modulus measurements, the effect of moisture condition for both tested concretes should be considered negligible.

To sum up, it should be stated that the impact of concrete moisture condition on measurements of its modulus of elasticity, as well as the magnitude of this effect, depends on the type of cement composite, particularly on its structural homogeneity and pore structure, as well as the type of test. Generally, the ultrasonic method used for dynamic modulus determination turned out to be markedly more sensitive to the moisture influence compared to the cyclic loading method used for static modulus determination. Nevertheless, this effect may not even occur at dynamic modulus measurements of concretes with a dense, homogeneous structure.

The above conclusions emphasize the importance of considering concrete moisture content not only during modulus tests but also when using equations to assess concrete secant static modulus following its dynamic value. The development of a reliable method to take into account the influence of concrete moisture in both tests and estimates of the elastic modulus requires further research, in particular extended to concretes of other compositions and other classes.

## Figures and Tables

**Figure 1:** Normal-weight coarse aggregate 4/16 mm was used for composite preparation.

**Figure 2:** Test specimens cured in water (**a**) and in air (**b**).

**Figure 3:** Cycles for the determination of stabilized secant modulus of elasticity (Method B): (**a**) according to EN 12390-13; (**b**) recorded for one NC1 specimen.

**Figure 4:** Testing equipment used for measurements of static secant modulus of elasticity: (**a**) a concrete cylinder under compression; (**b**) automatically controlled compressive testing machine.

**Figure 5:** Testing equipment used for measurements of ultrasonic pulse velocity.

**Figure 6:** Examples of normal-weight concretes after failure at compression: (**a**) Typical failure method; (**b**) typical fracture pattern.

**Figure 7:** Dynamic modulus (*E_d_*) as a function of ultrasonic pulse velocity (*V*), taking into account concrete moisture conditions (dried or wet) and concrete density (oven-dry or current).

**Figure 8:** Individual results of dynamic and static moduli measurements for NC1 dried and wet specimens tested at 3 years. Dashed lines indicate the level of average values.

**Figure 9:** Individual results of dynamic and static moduli measurements for NC2 dried and wet specimens tested at 3 years. Dashed lines indicate the level of average values.

**Figure 10:** Mean results of dynamic and static moduli measured on dried and wet specimens of lightweight concretes (based on [14]) and normal-weight concretes tested at 3 years.

**Table 1:** Composition of structural concretes to be tested in kg/m^3^.

Series	w/c	Coarse Aggregate 4/16 mm	Fine Aggregate 0/2 mm	Cement	Water	Superplasticizer
NC1	0.55	1140	570	377	208	0
NC2	0.37	1140	570	470	174	1.9

**Table 2:** Type of tests, number of cylinder specimens, age of concrete, and standard procedures.

Type of Test	Number of Cylinders	Age of Concrete	European Standard
Oven-dry density	3	28 days	EN 12390-7 [23]
Water-saturated density			
Compressive strength	6	28 days	EN 12390-3 [24]
Static modulus of elasticity	3	28 days	EN 12390-13 [7]
As-received density	3	3 years	EN 12390-7 [23]
Water-saturated density			
Oven-dry density			
Compressive strength	3	3 years	EN 12390-3 [24]
Static modulus of elasticity	3	3 years	EN 12390-13 [7]
Dynamic modulus of elasticity			EN 12504-4 [25]

**Table 3:** Mean values of basic concretes’ properties determined at 28 days.

Series	*f_cm_*, MPa	*E_c,s_*, GPa	*D_w_*, kg/m^3^	*D_d_*, kg/m^3^
NC1	42.9	25.0	2330	2220
NC2	59.5	30.1	2340	2290

**Table 4:** Mean values of basic concretes’ properties determined at the age of 3 years.

Series	*f_cm_*, MPa	*D_ad_*, kg/m^3^	*D_w_*, kg/m^3^	*D_d_*, kg/m^3^
NC1	51.6	2250	2340	2220
NC2	71.4	2300	2340	2290

**Table 5:** Values of secant modulus and strength measured at compression.

Concrete Designation	Cylinder Designation	Static Secant Stabilized Modulus of Elasticity, GPa				Compressive Strength, MPa	
		Dried Specimens		Wet Specimens			
		*E* *_c,si_*	*E* *_c,s_*	*E* *_c,si_*	*E* *_c,s_*	*f* *_ci_*	*f* *_cm_*
NC1	1	30.7	30.3	29.8	29.9	54.2	52.5
	2	30.4		29.4		53.1	
	3	29.9		30.6		50.2	
	3 *			30.5 *			
NC2	1	34.5	34.6	33.8	33.4	65.7	74.6
	2	35.3		32.6		80.7	
	3	34.1		33.8		77.5	
	3 *			33.7 *			

* Cylinders retested at different sensors locations.

**Table 6:** Measured values of *V*.

Concrete Designation	Cylinder Designation	Path Length, mm	Ultrasonic Pulse Velocity, m/s			
			Dried Specimens		Wet Specimens	
			*V* *_i_*	*V* *_m_*	*V* *_i_*	*V* *_m_*
NC1	1	294	3992	4005	4345	4311
	2	295	3966		4288	
	3	295	4058		4299	
NC2	1	299	4215	4181	4155	4203
	2	295	4245		4229	
	3	298	4084		4225	

**Table 7:** Estimated values of *E_d_*.

Concrete Designation	Cylinder Designation	Dynamic Modulus of Elasticity, GPa			
		Dried Specimens		Wet Specimens	
		*E* *_di_*	*E* *_dm_*	*E* *_di_*	*E* *_dm_*
NC1	1	31.8	32.1	37.7	37.1
	2	31.4		36.7	
	3	32.9		36.9	
NC2	1	36.6	36.0	35.6	36.4
	2	37.1		36.9	
	3	34.4		36.8	

## Data Availability

Data are contained within the article.
